# *Neisseria sicca* and *Corynebacterium matruchotii* inhibited oral squamous cell carcinomas by regulating genome stability

This article has been retracted.

**DOI:** 10.1080/21655979.2022.2078556

**Published:** 2022-06-23

**Authors:** Xin Shen, Bo Zhang, Xiaoyu Hu, Jia Li, Miaomiao Wu, Caixia Yan, Yutao Yang, Yan Li

**Affiliations:** a State Key Laboratory of Oral Diseases, National Clinical Research Center for Oral Diseases, West China Hospital of Stomatology, Sichuan University, Chengdu, Sichuan, China; b Department of Stomatology, Minda Hospital of Hubei Minzu University, Enshi, Hubei, China

**Keywords:** Periodontal negative-associated bacteria, OSCC, DNA damage response, inflammasomes, Anti-cancer

## Abstract

Periodontitis is a risk factor for the development of oral squamous cell carcinomas (OSCC). Both DNA damage response (DDR) and activation of inflammasomes induced by the microbiome might play important roles in the development of tumors, in relation to genome stability of tumor cells. Herein, we explored whether periodontitis negative-associated bacteria (*Neisseria sicca* and *Corynebacterium matruchotii*, namely called ‘PNB’), which were highly abundant in healthy populations, could inhibit OSCC by promoting genome stability. Firstly, a murine SCC-7 tumor-bearing model that colonized with PNB was designed and used in this study. Then, cyclin D1 was detected by immunohistochemistry. Levels of DDR, NLRP3 inflammasomes and pro-inflammatory cytokines in tumors were detected by RT-qPCR or Western blot. Immune cells in spleens were detected by immunohistochemistry or immunofluorescence. Finally, the anti-cancer activity of PNB was assessed *in vitro* using CCK-8 assays and flow cystometry. Compared with the control, PNB decreased tumor weights from 0.77 ± 0.26 g to 0.42 ± 0.15 g and downregulated the expression of Cyclin D1. PNB activated the DDR by up-regulating γ-H2AX, p-ATR, and p-CHK1. PNB activated NLRP3 inflammasome-mediated pyroptosis via increases of NLRP3, gasdermin D, and mRNA levels of apoptosis-associated speck-like protein, Caspase-1. PNB suppressed the inflammatory response by down-regulating mRNA levels of NF-κΒ and IL-6 in tumors as well as the populations of CD4+ T cells and CD206+ immune cells in spleens. PNB inhibited proliferation and promoted cell death of HSC-3 cells. In conclusion, *Neisseria sicca* and *Corynebacterium matruchotii* showed a ‘probiotic bacterial’ potential to inhibit OSCC by regulating genome stability.

## Highlights

- *N. sicca* and *C. matruchotii* inhibited the growth of OSCC
- Genome stability of OSCC was maintained by *N. sicca* and *C. matruchotii*
- Pro-inflammatory responses were suppressed by *N. sicca* and *C. matruchotii*

## Introduction

Oral squamous cell carcinomas (OSCC) account for over 90% of all the head and neck squamous cell carcinomas (HNSCCs) and OSCC patients have a 5-year survival rate < 50%, which cause a huge global health burden [1]. There are more than 350,000 new cases of OSCC and 175,000 deaths each year [2]. At present, the pathogenesis of OSCC is not clear. The interactions of microbial alterations and human cancers have been widely reported. In particular, some special periodontal bacteria are closely associated with the development of OSCC, such as *Porphyromonas gingivalis* and *Fusobacterium nucleatum* [3,4]. As for the dysbiosis of oral bacterial community, the probiotics are considered to have a potential activity of the anti-cancer. For example, the use of *Lactobacillus plantarum* for the treatment of OSCC was suggested [5,6]. The main treatment for OSCC is surgery, usually combined with radiotherapy and chemotherapy for the patients with advanced stages. However, radiotherapy and chemotherapy are more likely to be accompanied by the major side effects [7]. Moreover, microbial-based therapy has been proposed for the treatment of cancers [5]. Recently, advances in DNA sequencing technology have accelerated our understanding of the relationship between oral microbiome and OSCC. The promoting or suppressing effects of oral microbes on OSCC have been studied. In particular, the hypothesis that periodontitis-associated bacteria might contribute to OSCC has been widely analyzed [6,8]. Actually, our previous study identified periodontitis negative-associated bacteria, *Neisseria* and *Corynebacterium*, which are highly abundant in the healthy population [7]. However, whether those bacteria have influences on tumor regression and the related mechanisms are still unclear.

DNA damage surveillance mechanisms have important roles in the relationship between the microbiome and cancers [9]. The downregulation of damage surveillance mechanisms and the increases in genome instability might contribute to tumor progression [10]. To combat a variety of stresses in cells, a series of responses are activated by DNA damage, collectively known as DNA damage response (DDR). The DDR is a multi-step process that activates downstream responses, including DNA repair pathways involving p53 [11]. DNA damage signaling can be detected by modification of the phosphorylation of histone H2A variant (H2AX), ataxia-telangiectasia-mutated-and Rad3-related (ATR) and checkpoint kinase1 (CHK1), to maintain genome stability [12]. An intimate relationship between the cancer and DDR was proposed [12]. At an early stage of neoplastic lesions, the DDR is activated and is likely to induce anti-cancer networks in tissues and organs, such as the stomach, lung, colon, and breast [13]. When the damage is repaired effectively, the normal function of cells is restored; otherwise, the DDR triggers cell death, which has a potential anti-cancer effect [14,15]. The inactivation of DDR components during cancer development would contribute to malignant progression [15].

When a variety of exogenous stress and DNA damage signals attack, the host cells recruit PYD domains-containing protein (NLRP) inflammasomes to regulate immune responses to maintain genome stability. NLRP3 is widely activated by a variety of danger signals and it is positively associated with the reactive oxygen species, which are defined as mediators of DNA damage [16,17]. NLRP3 inflammasomes are protein complexes that consist of NLRP3, apoptosis-associated speck-like protein (ASC), and cysteinyl aspartate specific proteinase-1 (Caspase-1). The activation of NLRP3 inflammasomes leads to the maturation of caspase-1, which mediates the maturation of pro-inflammatory cytokines, such as IL-1β and IL-18 [18,19]. Another important role for caspase-1 is to cleave gasdermin D (GSDMD), which has been identified as a key executor of pyroptosis [20]. Pyroptosis is a type of lytic programmed cell death induced by inflammasomes. Recently, pyroptosis has been shown to have an anti-cancer activity via the recruitment of tumor suppressor immune cells [21]. Furthermore, tumors in the digestive tract are sensitive to the induction of pyroptosis [22]. It is unclear whether NLRP3 inflammasome-mediated pyroptosis is involved in the relationship between the periodontitis negative-associated bacteria and OSCC.

The core microbiota of periodontitis negative-associated bacteria, *Neisseria* and *Corynebacterium* [7], were highly abundant in the healthy population with an average relative abundance >5%. The sequences of representative Operational Taxonomic Units (OTUs) were blasted for alignment in the NCBI database to screen for the periodontitis negative-associated bacteria: *Neisseria sicca* (*N. sicca*) and *Corynebacterium matruchotii* (*C. matruchotii*). The aims of this study were to determine the ‘probiotic bacterial’ potential of *N. sicca* and *C. matruchotii*, to explore the effects of those bacteria on the regression of OSCC, and to determine whether those mechanisms were associated with genome stability. Thus, a murine SCC-7 tumor-bearing model that orally inoculated with *N. sicca* and *C. matruchotii* was used in our study. We found that an inhibitory effect of periodontitis negative-associated bacteria on OSCC was involved in the early activation of DNA damage signaling and NLRP3/GSDMD-mediated pyroptosis *in vivo* and the growth of tumor cells was inhibited by those bacteria *in vitro*. Improving the genome stability of tumor cells by oral probiotic microbiota might be the potential effective prevention and treatment strategies of OSCC.

## Materials and methods

### Bacteria

The core OTUs of different genera from periodontitis negative-associated bacteria were analyzed in our previous 16S RNA gene sequencing study [7] and the sequences of representative OTUs were blasted for alignment in the NCBI database to screen for periodontitis negative-associated bacteria (PNB): *N. sicca* and *C. matruchotii. N. sicca* (ATCC 29256) were preserved in the microbial strain bank of State Key Laboratory of Oral Diseases, Sichuan University, and *C. matruchotii* (ATCC 14266) were purchased from American Type Culture Collection. Those bacteria were grown overnight in Brain Heart Infusion broth under aerobic conditions at 37°C and were harvested in the exponential growth phase. According to the sequencing results of their relative abundance, the ratio of *N. sicca* and *C. matruchotii* was determined to be 3:2.

### Cell culture and treatment

The human HSC-3 and mouse SCC-7 cell lines were kindly provided by Prof. Qianming Chen (State Key Laboratory of Oral Diseases, Sichuan University). Both cell lines were cultured in DMEM (HyClone, USA) with 10% FBS (Gibco, Australia) at 37°C in a humidified cell incubator (Thermo Fisher Scientific, USA) with 5% CO_2_. Cells at 75% confluence were used for these studies. According a previous study [23], a MOI of 200 was selected for use in subsequent experiments to detect the viability and apoptosis of HSC-3 cells.

### Cell viability detection

A CCK-8 kit (Biosharp, China) was used to detect the viability of HSC-3 cells. At 8 h after co-infection with PNB, HSC-3 cells were washed three times with PBS (GIBCO, USA) and then were cultured for another 12 h with metronidazole (200 μg/ml) (Solarbio, China) and gentamicin (300 μg/ml) (Solarbio, China) in DMEM [24]. Those cells were seeded in 96-well plates at 3 × 10^3^ cells/well and cultured for 24, 48, 72, and 96 h. Ten μL CCK-8 solution was added to the medium for 2 h at room temperature and OD_450_ values were detected using a Varioskan Flash microplate reader (Thermo Fisher Scientific, USA).

### Analysis of dead and apoptotic cells

Dead and apoptotic rate of HSC-3 cells were detected by flow cytometry using an Annexin V-FITC/PI Apoptosis kit (Keygen Biotech, China). HSC-3 cells were seeded in six-well plates at 2 × 10^6^ cells/well. After 24 h of co-infection with PNB, HSC-3 cells were harvested and stained following the manufacturer’s protocol. Flow cytometry (Beckman FC500, USA) was used to detect the dead and apoptotic rate of HSC-3 cells.

### Animal model

The Ethics Committee of the West China Hospital of Stomatology, Sichuan University (WCCSIRB-D-2016-052) approved this study. *N. sicca* and *C. matruchotii* (PNB) were harvested in the exponential growth and centrifuged for 10 min at 4,000 × g and 4°C. PBS was used to wash the bacterial sediments for three times. Ten × 10^8^ colony forming units of PNB were mixed in 200 μL Carboxymethy Cellulose (CMC) (Solarbio, China) and were used for the bacterial colonization in animal experiments. BALB/c mice (8 weeks old, males) were purchased from Dossy Experimental Animals Co., Ltd (Chengdu, China). Those mice were housed in a specific pathogen-free environment and were randomized into two groups: one group was orally inoculated with PNB (P-, n = 5), while the other group was treated with CMC only and served as a control (Control, n = 5). All mice were fed with four mixed antibiotics (1 g/L ampicillin, 1 g/L metronidazole, 1 g/L neomycin, and 0.5 g/L vancomycin) (Solarbio, China) which were dissolved in the drinking water for 3 days before the bacterial colonization [25]. Colonization experiments were performed at one-day interval- after the antibiotic treatment. PNB in 2% CMC were applied into the oral cavity of each mouse for four times a week as previously described [26]. Two weeks later, 5 × 10^6^ SCC-7 cells suspended in 50 μL DMEM without FBS were injected into the sub-mucosa of the right cheek of each mouse [27]. Bacterial inoculations were continued for 3 weeks after which all mice were euthanized. Tumor volumes and weights were evaluated. Tumor volumes were determined using the following formula: Tumor volume (mm^3^) = (minimum diameter)^2^ × (maximum diameter)/2 [28].

### Histopathology, immunohistochemistry, and immunofluorescence

After paraffin-embedding of the tumors, serial sections were cut, then deparaffinized and rehydrated, after which they were stained with hematoxylin-eosin (HE) and analyzed by immunohistochemistry (IHC). IHC and immunofluorescence (IF) were also used to analyze the sections of spleen. According to the manufacturer’s protocol, the following antibodies were used: cyclin D1 (1:500), γ-H2AX (1:200), CD4 (1:500), CD8 (1:500), CD206 (1:500), all purchased from Cell Signaling Technology, USA. Antibodies to NLRP3 (1:100, Abmart, China) and GSDMD (1:1,000, Abcam, USA) were also used. Secondary antibody IgG (1:10,000, solelyBio, China) and Alexa Fluor 488 (1:100, Servicebio, China) were used to detect bound primary antibodies according to the manufacturer’s protocol. IHC staining of cyclin D1, γ-H2AX and CD206 were scored by the proportion of highly positive cells, while NLRP3, GSDMD, CD4, and CD8 were scored by the mean IHC scores (0: negative, 1: low positive, 2: positive, 3: high positive) using Image J software (version 1.8.0_172, USA).

### Analysis of micro-scale computed tomography (μCT)

High-resolution μCT (Viva CT40, Scanco Medical, Bassersdorf, Switzerland) was used to scan the hemi-mandibles of mice. The parameters of μCT were at 45 keV with a 10 μm isotropic voxel size for data analysis. The distances between the cemento-enamel junction and the alveolar bone crest in medium region of the first and second molar teeth were evaluated to describe the alveolar bone loss (mm). Three-dimensional reconstructions were performed using a set of 400 slices.

### RNA isolation and real-time qPCR

TRIzol (Invitrogen, USA) was used to isolate and extract the total RNAs. The concentration and purity of RNAs were quantified by spectrophotometry (Applied Biosystems, USA). Reverse transcription of RNAs into cDNAs was performed using a PrimeScript RT Reagent Kit with gDNA Eraser RR047A (Takara Bio, Japan). Real-time polymerase chain reactions were performed using a Step One Plus Real-time PCR System (Applied Biosystems, USA). All primers used for gene assays are shown in Table 1, which were designed by Primer-BLAST online (https://www.ncbi.nlm.nih.gov/tools/primer-blast/) and produced by Biochemical Bioengineering (Shanghai, China). The ^2–ΔΔ^CT method was used for the relative quantitative analysis of mRNA concentrations. GAPDH was served as the internal control.

**Table 1.** List of primer sequences used for real-time PCR.

Name	Forward primer	Reverse primer
P53	5’- TGGAAGGAAATTTGTATCCCGA −3’	5’- GTGGATGGTGGTATACTCAGAG −3’
γ-H2AX	5’- CTTCAGTTCCCTGTAGGCC −3’	5’- GATCTCGGCAGTGAGGTAC −3’
ATR	5’- ACCAAAAGGAGGTAAGGTCAACA −3’	5’- AGGACGCTACAGCCAGAGTA −3’
CHK1	5’- ATGAAGCGGGCCATAGACTG −3’	5’- GGATATGGCCTTCCCTCCTG −3’
NF-κΒ	5’- CAAAGACAAAGAGGAAGTGCAA −3’	5’- GATGGAATGTAATCCCACCGTA −3’
IL-6	5’- CTCCCAACAGACCTGTCTATAC −3’	5’- CCATTGCACAACTCTTTTCTCA −3’
NLRP3	5’- ATGTGAGAAGCAGGTTCTACTC −3’	5’- CTCCAGCTTAAGGGAACTCATG −3’
ASC	5’- ACAATGACTGTGCTTAGAGACA-3’	5’- CACAGCTCCAGACTCTTCTTTA −3’
Caspase-1	5’- AGAGGATTTCTTAACGGATGCA −3’	5’- TCACAAGACCAGGCATATTCTT −3’
IL-18	5’- AGACCTGGAATCAGACAACTTT −3’	5’- TCAGTCATATCCTCGAACACAG −3′
IL-1β	5’- CAACTGTTCCTGAACTCAACTG −3’	5’- GAAGGAAAAGAAGGTGCTCATG −3′
GAPDH	5’-GTGTTTCCTCGTCCCGTAGA-3’	5’-AATCTCCACTTTGCCACTGC-3’

### Western blot

Samples for western blotting were prepared using a Total Protein Extraction Kit (Signalingway Antibody, USA) following the manufacturer’s instructions. Protein samples were mixed with 5 × SDS buffer (Beyotime, China), and then denatured prior to separation on 10% SDS-PAGE gels. After transferring to membranes and blocking, the following antibodies were used: anti-γ-H2AX (1:1,000), anti-p-ATR (1:1,000), anti-p-CHK1 (1:1,000) and anti-p53 (1:10,000), all obtained from Cell Signaling Technology, USA. Goat anti-Mouse/Rabbit IgG Secondary Antibodies HRP Conjugated (1:8,000, Signalingway Antibody, USA) were used to detect bound primary antibodies. α-tubulin (1:6,000, HuaAn Biotechnology, China) was used as an internal control. Image J software (version 1.8.0_172, USA) was used for image analysis.

## Statistical analysis

SPSS (version 24.0, IBM Corporation, USA) was used for statistical analyses. Data were shown as means ± SEM. Unpaired Student’s t-tests were used to compare differences between the two groups. P value < 0.05 was considered significant.

## Results

### Effects of PNB on tumor growth in SCC-7 tumor-bearing mice

PNB might have influences on the regression of OSCC. Thus, a murine SCC-7 tumor-bearing model that was orally inoculated with PNB was used in our study, to evaluate the effect of PNB on the growth of OSCC. As shown schematically in Figure 1(a), the animal experimental protocol lasted for 42 days. Compared with the control, there was a decreasing trend of tumors in the P- group, from 0.43 ± 0.11 cm^3^ to 0.27 ± 0.06 cm^3^ in average tumor volume at the endpoint week (at 42 days) (Figure 1(b), p > 0.05). And the average tumor weight was 0.42 ± 0.15 g in the P- group, which was 47% lower than the control group, which was 0.77 ± 0.26 g. (Figure 1(c,d), p > 0.05). Although a significant decreasing trend was induced by PNB, the tumor volumes and weights were not significantly different between the two groups. Thus, we wanted to know how PNB affected histological changes of tumors. Hematoxylin-eosin staining showed that tumor vascular proliferation was decreased by PNB (indicated by the black arrows, Figure 1(e)). Moreover, to determine whether there was an inhibitory role of PNB on tumor growth, cyclin D1 expression was measured. Compared with the control, cyclin D1 was significantly decreased about 50% in the P- group (Figure 1(e), p < 0.05). Finally, to verify whether PNB showed an inhibitory effect on alveolar bone loss in SCC-7 tumor-bearing mice, μCT was used. Compared with the control, the alveolar bone loss was significantly decreased by PNB, from 0.42 ± 0.03 mm to 0.21 ± 0.02 mm (Figure 1(f), p < 0.05).

**Figure 1.** Effects of PNB on tumor growth in SCC-7 tumor-bearing mice. (a) Overview of the experimental protocol of SCC-7 tumor-bearing mice that orally inoculated with PNB. Antibiotic treatments were represented by the yellow squares, and orally inoculated with PNB was represented by the blue squares. (b) Tumor volumes measured at the end of the experiment. (c) Tumor weights detected at the end of the experiment. (d) Gross appearance of tumors. (e) Representative immunohistochemical staining for Cyclin D1 in tumor tissues (high positive cells were indicated by the black arrows). Scale bars, 50 μm. (f) Alveolar bone loss was shown by the red areas in three-digital reconstructions (3D) and the distances between two horizontal lines (blue and red) in sagittal slice views (2D). Scale bars, 1 mm. Control, SCC-7 tumor-bearing mice that orally inoculated with CMC (n = 5); P-, SCC-7 tumor-bearing mice that orally inoculated with PNB (n = 5). Data were represented as means ± SEM. *p < 0.05.

### ATR-CHK1 signaling was activated by PNB in SCC-7 tumors

At an early stage of tumors, DNA damage signaling is activated by the phosphorylated protein cascades and is likely to induce anti-cancer networks. Moreover, periodontitis-associated bacteria have been identified as ‘bad bacteria’ to increase genome instability of OSCC []. Thus, we wanted to determine whether PNB could promote the genome stability of OSCC by up-regulating DNA damage signaling. The accumulation of γ-H2AX is a signature event in DNA damage signaling. The number of cells highly positive for γ-H2AX (by two-fold or more) was significantly upregulated by PNB in tumor tissues (Figure 2(a), p < 0.01). Next, the factors involved in the DNA damage repair pathway, such as ATR/CHK1/p53 signaling, were evaluated by detecting proteins using Western blots. Compared with the control, the expression levels of p-ATR (p < 0.05) and p-CHK1 (p < 0.05) were increased dramatically, while the level of p53 (p > 0.05) was slightly upregulated in the P- group with no significant difference (Figure 2(b)). Indeed, the mRNA levels of γ-H2AX, ATR and CHK1 were significantly upregulated by PNB (Figure 2(c), p < 0.05). However, there was no significant difference between the two groups in the mRNA expression level of p53 (Figure 2(b), p > 0.05).

**Figure 2.** ATR-CHK1 signaling was activated by PNB in SCC-7 tumors. (a) Representative immunohistochemical staining for γ-H2AX in tumor tissues (high positive cells were indicated by the black arrows). Scale bars, 50 μm. (b) Proteins of DNA damage repair signaling. α-Tubulin was used as a loading control. Western blot bands were quantified. (c) Histogram of the relative mRNA (fold change) expression level of genes involved in DNA damage repair signaling. Data were representative of three independent experiments. Data were represented as means ± SEM. *p < 0.05, **p < 0.01.

### NLRP3/GSDMD-mediated pyroptosis was upregulated by PNB in tumors

When bacteria and DNA damage signals attack, the host cells recruit NLRP3 inflammasomes to regulate cytokines and to promote genome stability by pyroptosis. To determine how PNB affect the NLRP3 inflammasome-mediated pyroptosis, the mRNA and protein levels of NLRP3 inflammasomes(NLRP3, ASC, and Caspase-1), cytokines (IL-1β and IL-18), and GSDMD were detected by RT-qPCR or IHC. As shown in Figure 3(a), the expression of NLRP3 was significantly increased in the P- group (p < 0.05). The key protein involved in pyroptosis, GSDMD, was also significantly upregulated by PNB (p < 0.05). The mRNA level of NLRP3 inflammasomes expressed in tumor tissues was detected. Compared with the control, the mRNA levels of ASC (p < 0.05) and Caspase-1 (p < 0.05) were significantly upregulated in the P- group, while the mRNA level of IL-1β (p <0.05) was significantly decreased (Figure 3(b)). There was no significant difference in the mRNA level of NLRP3 or IL-18 between the two groups (Figure 3(b), p > 0.05).

**Figure 3.** NLRP3/GSDMD-mediated pyroptosis was upregulated by PNB in tumors. (a) Representative immunohistochemical staining for NLRP3 and GSDMD in tumor tissues (positive cells were indicated by the black arrows). Scale bars, 75 μm. (b) Histogram of the relative mRNA (fold change) expression levels of NLRP3 inflammasomes factors. Data were representative of three independent experiments. Data were represented as means ± SEM. *p < 0.05, **p < 0.01.

### The inflammation level was suppressed in tumors and spleens by PNB

Increasing levels of inflammatory cytokines have been found in OSCC. Our previous study showed that periodontitis-associated bacteria contributed to the inflammatory responses in the SCC-7 tumor-bearing model, but how PNB affect the inflammation of OSCC is unclear. Changes in the three types of immune cells in the spleens (CD4+, CD8+ T cells, and CD206+ cells) and pro-inflammatory cytokines in tumors (NF-κB and IL-6) were detected. Levels of CD4+ T and CD206+ cells (M2 macrophages) were decreased by PNB (Figure 4(a,b), p < 0.05). However, CD8+ T cells were slightly decreasing with no significant difference between the two groups (Figure 4(a,b), p > 0.05). Regarding the levels of pro-inflammatory cytokines in tumors, the relative mRNA levels of NF-κB and IL-6 were downregulated by PNB, compared with the control (Figure 4(c), p < 0.05).

**Figure 4.** The inflammation level was suppressed in tumors and spleens by PNB. (a) Representative immunohistochemical staining for CD4+ and CD8+ T cells, and immunofluorescence staining for CD206+ cells. Positive expression cells were indicated by the white arrows. White pulp (W) and red pulp (R) of the spleen were shown. Scale bars, 100 μm. (b) Histograms showing the mean IHC scores for CD4+ and CD8+ T cells (left) of images shown in panel A and the % of IF scores for CD206+ cells (right) of images shown in panel A. (c) Histogram of the relative mRNA (fold change) expression level of pro-inflammatory factors in the tumors. Data were represented as means ± SEM. *p < 0.05.

### The growth of HSC-3 cells was inhibited by PNB

An inhibitory effect of PNB on OSCC was determined *in vivo*, but it is not clear how those bacteria influence the activity of tumor cells *in vitro*. Thus, a co-infection of PNB with HSC-3 cell model was assessed using CCK-8 assays. Compared with the control, 8 h of co-infection with PNB significantly reduced the growth of HSC-3 cells at 24, 48, 72, and 96 h (Figure 5(a), p < 0.05). Moreover, the rate of cell death in HSC-3 cells was dramatically increased from 0.50 ± 0.15% to 4.85 ± 1.15% (Figure 5(b), p < 0.05). However, the cell apoptotic rate was increased with no statistically significant level (Figure 5(b), p > 0.05).

**Figure 5.** The growth of HSC-3 cells was inhibited by PNB *in vitro*. (a) The viability of HSC-3 cells with 8 h post-infection was determined using the CCK-8 assay at 24, 48, 72, and 96 h. (b) HSC-3 cells with 24 h post-infection stained with Annexin V-FITC/PI were analyzed by flow cytometry. Dead cells were represented by the Annexin V-FITC negative and PI positive, while apoptotic cells were represented by the Annexin V-FITC positive. Control, HSC-3 cells were co-cultured with PBS; P-, HSC-3 cells were co-infected with PNB. Data were means ± SEM. *p < 0.05. Results were representative of three independent experiments.

In summary, the potential mechanisms of the inhibitory effect of *N. sicca* and *C. matruchotii* on the regression of OSCC were described in this study. *N. sicca* and *C. matruchotii* restrained the development of OSCC by maintaining genome stability, mainly including the activation of DNA damage signaling by upregulating the phosphorylation of ATR and CHK1 as well as by activating NLRP3/GSDMD-mediated pyroptosis in tumor cells. The levels of inflammatory cytokines were suppressed by *N. sicca* and *C. matruchotii* in the tumor microenvironment, including NF-κΒ and IL-6 in the tumor and CD4+ and CD206+ T cells in the spleen.

## Discussion

Several research studies have proposed that oral microbiome is associated with the development of OSCC and oral microbial dysbiosis is present in OSCC [8]. Compared with the healthy controls, the abundance of *Neisseria* is decreasing in the HNSCC patients [29,30] and *Neisseria* are associated with reducing the risk of oral cancers [31]. Furthermore, an inhibitory ability of *Neisseria* on the proliferation of OSCC cells was observed *in vitro* [32]. On the other hand, Hayes *et al*. reported that a greater abundance of the genera *Corynebacterium* is associated with a decreasing risk of the HNSCCs [31]. However, evidence of the role of *Neisseria* and *Corynebacterium* in the development of OSCC is still limited. The evidence above indicates that the genera *Neisseria* and *Corynebacterium* might have a negative correlation with OSCC development and the potential anticancer properties. Consistent with those results, a mixture of *N. sicca* and *C. matruchotii* inhibited the growth of HSC-3 cells *in vitro* and contributed to tumor regression in SCC-7 tumor-bearing mice *in vivo* in our study. Of course, it is necessary to increase sample sizes to obtain the significant results in the volumes and weights of tumors. The main function of cyclin D1 is to promote cell proliferation and it has been recognized as a proto-oncogene [33]. The overexpression of cyclin D1 commonly has been observed in OSCC [34]. Periodontitis-associated bacteria, such as *P. gingivalis* and *F. nucleatum*, might upregulate the expression of cyclin D1 in OSCC [8]. On the contrary, some anticarcinogens can inhibit the proliferation of oral cancer cells by decreasing of cyclin D1 levels [35]. Our results showed that cyclin D1 expression was decreased by *N. sicca* and *C. matruchotii*, which might have an opposite effect of periodontitis-associated bacteria. This indicates that periodontitis negative-associated bacteria might have a suppressing effect on oral cancer. However, there is more evidence that needs to be confirmed the potential role of periodontitis negative-associated bacteria in OSCC.

DDR has important roles in maintaining genome stability and their components frequently are inactivated in tumors. DDR might be activated in the early stage of tumor development, leading to blockade of the cell-cycle to repair DNA damage and thereby limiting tumor progression, such as tumors that occur in the lungs, colon, and breast [13]. If DNA damage is not accurately repaired, DDR triggers cell death in tumors, which has a potential anti-cancer effect [14,15]. The inactivation of DDR might promote tumor development [12]. In our study, ATR-CHK1 signaling was activated by *N. sicca* and *C. matruchotii* in SCC-7 tumor-bearing mice, and the cell death of HSC-3 was increased by those bacteria *in vitro*. Consistent with the potential anti-cancer effect of the DDR as described above, *N. sicca* and *C. matruchotii* might upregulate DDR and induce tumor cell death to help OSCC regression.

The crosstalk between the mechanisms of cell death and anti-cancer immunity has been proposed in a few studies, including ferroptosis, necroptosis, and pyroptosis [21]. A variety of the mechanisms of cell death might be regulated by NLRP3 inflammasomes. In response to many stimuli, NLRP3 inflammasomes act as ‘the Vanguard’. Activation of NLRP3 inflammasomes triggers the maturation of caspase-1, which induces expression of pro-inflammatory cytokines such as IL-1β and IL-18 [36]. In addition, activated caspase-1 might cleave GSDMD to induce pyroptosis [20]. Recently, two studies reported that tumor cells might recruit immune cells for tumor suppression by pyroptosis, which could play a role of anti-cancer. If less than 15% of tumor cells undergo pyroptosis, it would be sufficient to clear all the xenograft in mice [37,38]. On the other hand, owing to the activation of pyroptosis, many inflammatory cytokines are released, which might contribute to tumor development [39]. Pyroptosis has both tumor promoting and tumor suppressing roles that might depend on the environment. Our results showed that periodontitis negative-associated bacteria activated NLRP3 inflammasomes and GSDMD, which might induce pyroptosis and tended to have an anti-cancer role in OSCC.

It lasted a long time in an inflammatory condition before tumor formation, approximately 15 ~ 20% of inflammatory tumors [40]. Increasing levels of inflammatory cytokines are involved in OSCC, such as NF-κΒ [41]. Over-expression of NF-κB and IL-1β are associated with the advanced stage tumors and a poor survival rate of the OSCC patients [42,43]. IL-1β plays a key role in carcinogenesis due to its importance as a critical downstream mediator of inflammation [44,45]. Similarly, the elevated expression of IL-6 is associated with tumor progression [46]. In our study, the mRNA levels of NF-κΒ, IL-6 and IL-1β were downregulated by *N. sicca* and *C. matruchotii*, which might play an anti-inflammatory role in OSCC. A low level of immune infiltration in the spleen was also observed, including CD4+ T cells and CD206+ cells (M2 macrophages) of mice that were orally colonized with *N. sicca* and *C. matruchotii*. M2 macrophages might play important roles in regulating the proliferation and invasion of OSCC. Notably, a high number of M2 macrophages are significantly correlated with a poor prognosis in cancer [47]. Thus, a low number of M2 macrophages might have the opposite effect on OSCC. *N. sicca* and *C. matruchotii* decreased the number of M2 cells, which might have a protective effect on OSCC in our study. The role of CD4+ T cells has not been well clarified. On the one hand, CD4+ T cells are required for efficacious antitumor immunity [48], and all CD4+ T cells in the tumor were found to be significantly reduced in oral cancer patients [49]. However, a significant increase of CD4+ T cells was observed in peripheral blood mononuclear cells in OSCC patients [50–53]. It indicated that a lower population of CD4+ T cells in the peripheral blood might contribute to tumor regression. In our study, CD4+ T cells in the spleen were decreased by *N. sicca* and *C. matruchotii*, which might have a protective effect in OSCC.

## Conclusions

In conclusion, this study provided new insights into the role of oral microbiome in tumor regression, especially the inhibitory effects of periodontitis negative-associated bacteria, such as *N. sicca* and *C. matruchotii*, on OSCC. Particularly, the activation of ATR-CHK1 signaling and NLRP3/GSDMD-mediated pyroptosis induced by *N. sicca* and *C. matruchotii* have potential effects on promoting the genome stability of OSCC. However, it is not clear whether the effects of periodontitis negative-associated bacteria are directly focused on tumors or are mediated by the intestinal microbial dysbiosis. Thus, the inhibitory mechanisms of *N. sicca* and *C. matruchotii* on OSCC need to be verified, through the detection of changes in the oral or gut bacterial community in the future. The potential applications of *N. sicca* and *C. matruchotii* for the prevention and treatment of oral cancers are worth further investigation.
